# The Perspectives of Surrogates and Healthcare Providers Regarding SDM (Shared Decision-Making)

This article has been retracted.

**DOI:** 10.1155/2023/6251492

**Published:** 2023-02-11

**Authors:** Qing Lu, Juan Ji, Xiaoyan Lu, Qionghua Yin, Yiqun Yang

**Affiliations:** ^1^Department of Intensive Care Unit, The First Affiliated Hospital of Soochow University, Suzhou, China; ^2^Department of Radiotherapy, The First Affiliated Hospital of Soochow University, Suzhou, China; ^3^Nursing Department, The First Affiliated Hospital of Soochow University, Suzhou, China

## Abstract

The purpose of this paper is to explore the attitudes of surrogacy and medical service providers toward SDM and to identify the barriers and promoters of SDM in this population. To this end, we conducted a qualitative study of surrogacy and medical service providers in the First Affiliated Hospital of Soochow University using semistructured interviews. Thirty participants (11 agents, 12 ICU physicians, and 7 ICU nurses) were interviewed. The three stakeholders showed different attitudes toward SDM. They reported barriers to SDM, including insufficient cognition of decision-makers, high expectations, negative psychological experiences, previous decision-making experiences, excessive workload, heavy financial burden, and lack of decision AIDS. They reported facilitators of SDM, including trust, effective communication, decision support, value clarification, outcome commitment, and continuous service. This study explored the different attitudes of the three stakeholders and identified various barriers and facilitators of SDM. It highlights the need to develop localised decision AIDS and to involve agents and nurses more in the decision-making process. Therefore, this paper identifies barriers and facilitators of SDM in this population. In addition, the study identified various barriers and facilitators to SDM and highlighted the need to develop localised decision AIDS and involve agents and nurses more in the decision-making process. Finally, the barriers and facilitators of SDM are established. The paper also shows that the development of localized decision AIDS and greater involvement of agents and nurses in the decision-making process are integral to good treatment outcomes.

## 1. Introduction

Because of the development of society and medicine, people's awareness of health protection and participation in the process of disease diagnosis and treatment are constantly improving. At the same time, it also promotes the concept of shared decision (SDM). After more than 40 years of research and clinical practice, shared decision-making has become quite mature in developed countries such as Europe and the United States. In 2016, the ethics committees of the American College of Critical Care Medicine (ACCM) and the American Thoracic Society (ATS) recommended the use of SDM to define overall care goals in the ICU. However, at present, family decision-making participation, patient values, and treatment intention are paid less attention in ICUs in China. All these indications indicate that the feasibility and effectiveness of SDM in ICU are the current problems that need to be solved.

## 2. Background

Stakeholder management is a common expression in business today, but the concept and its practical implications for how stakeholder relationships should be managed and how they should be managed remain at the center of lively discussions across multiple disciplines, notably business ethics, management theory, corporate law, and organizational theory. Freeman defines stakeholders as follows: “In a narrow sense, stakeholders are all identifiable groups or individuals on which an organization depends for survival, sometimes referred to as key stakeholders: shareholders, employees, customers, suppliers, and key government agencies. At a broader level, however, a stakeholder is any identifiable group or individual who can influence or be influenced by an organization's performance in terms of products, policies, and work processes. In this sense, public interest groups, protest groups, local communities, government agencies, trade associations, competitors, trade unions and the media are all organisational stakeholders.” Colle De S., [1].

The implementation of shared decision-making (SDM) in the intensive care unit (ICU) embodies the ethical principles of autonomy, nonharm, benefit, and justice [2] orative process that allows patients or their surrogate decision-makers (surrogates) and healthcare providers to make decisions together on the basis of the best scientific evidence available and patients' values, goals, and preferences [3].

In 2016, the American College of Critical Care Medicine (ACCM) and the American Thoracic Society (ATS) ethics committee recommended the use of SDM to define overall care goals which include limiting or withdrawing from life-prolonging interventions and making preference-sensitive treatment decisions [3]). The default SDM approach includes three key stages: information exchange, deliberation, and treatment decision. A well-functioning ICU team comprising ICU physicians, ICU nurses, and other members is critical to the SDM process [4]. It greatly influences improvement of patient outcomes, increase of medical satisfaction, and reduction of medical costs and moral distress of surrogates [5–7].

However, patients' wishes and preferences are not respected, and the prognosis and treatment risks are not discussed in detail; the SDM approach is seldom adapted in the ICU. Scheunemann et al. found that physicians considered patients' values and preferences while making treatment recommendations in only 20 out of 244 conferences (8.2%) [5]. Kruser et al. found that ICU physicians invite family members to participate in SDM only when available medical treatments fail to achieve physiologic goals [8]. These peculiarities of the ICU workplace culture and practice style bring profound challenges to the implementation of SDM. Patients' families and friends assume the role of surrogates while being unsure of the preferences and wishes of coma patients. Therefore, in circumstances wherein the patient cannot be directly involved in treatment decision-making, consulting surrogates for SDM presents with distinct psychological, ethical, and communication challenges. Therefore, a better understanding of barriers and facilitators associated with the implementation of SDM is needed.

Although several factors affecting ICU SDM have been identified by researchers, such as patient/family willingness to participate in the decision-making process, staff expertise, and lack of time, in terms of previous studies, few researchers have explored barriers and facilitators from different SDM stakeholder groups in current ICU care [9, 10]. In addition, due to the participation of family decision-making in ICUs in China, patients' values and treatment intention are less important. To clarify the feasibility and effectiveness of ICU SDM is a problem that needs to be solved at present. Therefore, this study is aimed at exploring the perceptions of SDM among surrogates and healthcare providers (physicians and nurses) and at identifying barriers and facilitators of SDM in these individuals.

## 3. Methods

### 3.1. Study Design and Setting

We conducted a qualitative study using semistructured interviews of surrogates and healthcare providers from July 2020 to December 2020 at Suzhou University attached first hospital, which is a large tertiary center and teaching hospital. We chose a qualitative approach rather than a survey. This is to get a deeper understanding and to get the personal views of the participants. Since the need for SDM may be greater between surrogators and healthcare providers in patients with hospital stays longer than 3 days, surrogators were interviewed 3 days after admission [11]. SDM among the three stakeholder groups (physicians, nurses, and surrogators) in the ICU usually occurs (1) during daily multidisciplinary meetings attended primarily by the ICU physician and surrogators, (2) during regular family meetings where the presence of the ICU nurse is preferred but not required, and (3) if it is done in a relatively informal setting. The interview location will be at the bedside [12].

The local institutional review board approved this study. All participants provided written consent.

### 3.2. Participants

In order to obtain more objective and unbiased findings, three groups of participants recruited from a comprehensive ICU were interviewed: doctors, nurses (healthcare providers), and surrogates. Agents older than or 18 years old (authorized for the study), who were also the primary caregivers of inpatients, were selected to participate in face-to-face interviews. All substitutes reported discussing treatment goals, treatment-related risks, and possible outcomes for hospitalized patients with their healthcare provider prior to the interview. Healthcare providers include cases assigned to ICU inpatients.

### 3.3. Sampling

Thirty eligible participants (11 surrogates, 12 ICU physicians, and 7 ICU nurses) were interviewed. Although the sampling was based on convenience, we included as many demographic and professional characteristics as possible to ensure the authenticity of the study results. The study included surrogate mothers of different ages, genders, and relationships with patients. Again, we include healthcare providers of different ages, genders, job titles, and work experience.

### 3.4. Data Collection

The whole interview process of all interviewees is conducted in a private room by themselves, and the interview lasts 30-45 minutes. The interviews explored three themes related to the SDM domain framework (status quo, attitudes, barriers, and facilitators) [13]. According to the feedback from two pilot tests, we adjusted the interview outline to reduce medical jargon. All interviews were conducted by the same researcher (LQ). The researcher was trained in conducting interviews and performing interview analysis. The researcher had not conducted qualitative work on this topic before with the same interviewees. This is because we wanted to preserve the fact that at the beginning of the interview, the researchers introduced respondents to the concept of SDM to ensure that they had a clear understanding of the topic before the interview. This also ensures that they will not be forced to incorporate previous concepts. At the end of the interview, respondents were asked to complete a demographic survey. The interview was recorded. Data collection continues until theoretical adequacy is reached.

### 3.5. Data Analysis

Two researchers (LQ, JJ) used qualitative content analysis to summarize text responses from 11 agents and 19 healthcare providers [14]. Each researcher independently reviewed the notes word for word, highlighting specific words that seemed to capture key concepts of SDM among respondents and jotting down the main impressions and ideas used to develop the code. The researchers then discussed the emerging code, grouped them to reach consensus, and organized the themes to create meaningful clusters. After the first five transcripts were coded to determine the coding scheme, the agreed codes and themes were systematically applied to all transcripts. Themes, their descriptors, and representative citations were presented to the respondents and reviewed with them to solicit their opinions on whether these aspects correctly reflected their views on SDM.

## 4. Results

In total, 30 participants including 11 surrogates (Table 1) and 19 healthcare providers (12 ICU physicians and 7 ICU nurses; Table 2) were interviewed; there were no drop-outs. Among the participants, 8/11 surrogates and 6/19 healthcare providers were men. The mean age of surrogates and healthcare providers was 44.1 years (SD (standard deviation): 9.9 years) and 34.8 years (SD: 6.0 years), respectively. Notably, 5/11 patients were hospitalized for a medical condition, 4/11 underwent a planned surgery, and 2/11 underwent an emergency surgery. The median work experience of the 12 ICU physicians was 11 years (IQR (interquartile range): 5.0–28.0), whereas the corresponding statistic for the seven ICU nurses was 9 years (IQR: 2.0–22.0).

The data analysis was divided into 16 categories, and three themes were obtained: (1) different attitudes toward SDM, including the supportive attitude of doctors, the inconsistent attitude of nurses, and the contradictory attitude of agents. The specific content can be viewed in Table 3. (2) The obstacles of SDM, that is to say, the decision-makers have insufficient cognition, high expectation, negative psychological experience, existing decision-making experience, excessive workload, heavy economic burden, and lack of decision-making AIDS. The specific content can be viewed in Table 4. (3) The promoting factors of SDM are trust, effective communication, decision support, value clarification, outcome commitment, and continuous service. The specific content can be viewed in Table 5.

### 4.1. Theme 1: Different Attitudes toward SDM

When asked about decision-making process and SDM, different stakeholder groups showed different attitudes (Table 3). Physicians argue that the notion that the health care system has somehow evolved into a “patient-centered” approach to medicine has caught on. Internists encourage agents to participate in SDM and believe that they can make treatment decisions that are in the best interest of their patients through mutual consultation. They also point to the need to modify the decision-making process to meet the different needs of agents, especially as some agents prefer to leave the final decision to the physician.

In addition, with the increasing call for “patient participation,” nurses reported being constantly aware of the need for patients or their surrogates to participate in the decision-making process and witnessing the gradually increasing popularity of the concept of SDM. However, some nurses were skeptical about the necessity and effectiveness of the implementation of SDM and reported being concerned about the increase in the consumption of manpower and material resources associated with the implementation of SDM in clinical practice.

Surrogates believed that SDM would help them stay informed about different treatment plans and make a relatively clear decision; this would in turn reduce their psychological pressure. However, the premise of SDM was that surrogates perceive the need of SDM. A few surrogates expressed hesitation to participate in the decision-making process and feared that their involvement in the decision-making process will only interfere with physicians' work.

### 4.2. Theme 2: Barriers of SDM

We identified seven barriers of SDM in this theme (inadequate cognition of decision-makers, high expectation, negative psychological experience, previous decision-making experience, excessive workload, financial burden, and lack of decision aids). First, because of lack of parity in disease knowledge between physicians and patients, a part of the surrogates fell into a “physicians know the best” and “families with inadequate knowledge” category. They thought physicians do not want families to interfere in the treatment or be questioned. They felt that doing so may harm physicians' professional identity or may be perceived as a reflection of mistrust or lack of respect toward the physician. At the same time, some surrogates had unreasonably high expectations of the psychological recovery of the patients after the treatment; therefore, they focused only on the results without comprehensively considering other aspects of the treatment and its outcomes. Their judgments were often not purely rational and were driven by strong emotions. Overly optimistic expectations of surrogates promoted excessive use of invasive treatments and delayed palliative care for terminally ill patients.

Surrogates' psychological experiences of shock and worry and previous negative decision-making experiences also hindered the implementation of SDM. These strong emotions impaired their ability to process information, deliberate, and make trade-offs. In the absence of the patient, the choice of treatment should consider what the will and preference of the patient would have been. Some surrogates showed lack of readiness with making a choice within a short period of time, and therefore, they would seek help from physicians and choose the plan recommended by them. Some surrogates were too dependent on physicians, which was not conducive to the implementation of SDM. Besides, heavy economic burden of the treatment on family members was the most obfuscating and conflicting aspect affecting the decision-making process. Many surrogates found themselves in a dilemma while making a decision because of economic reasons. Particularly with making end-of-life decisions, life support treatment had to be discontinued due to the critical economic condition of the surrogates who could no longer afford the treatment expenses.

Healthcare providers reported that heavy work load did not allow them enough time to assess whether the ongoing treatment was still in line with patients' best interests or wishes. The daily workload of healthcare providers was high, and the time it would take to share decisions with each surrogate would further increase their work burden. Besides, decision aids are also an important factor affecting the implementation of SDM. Decision aids are effective means to promote surrogates' participation in the decision-making process; they help surrogates reach a decision after careful consideration of both their and patients' perspectives. However, ICUs of domestic hospitals lacked the tools that are typically provided by healthcare providers to help surrogates participate in SDM, and the effectiveness of a few decision aids introduced from abroad was unverified.

### 4.3. Theme 3: Facilitators of SDM

We identified 6 facilitators of SDM within this theme (trust, effective communication, decision support, value clarification, outcome commitment, and continuous service; Table 5). Both surrogates and healthcare providers believed that trusting in each other will make the decision-making process easier, particularly in the emergency situations. In the acute ICU setting, the stakeholders needed to establish agreement promptly for curing patients. Many physicians said that trust was based on the professional skills and control of the patient's condition. Meanwhile, surrogates viewed trust as one of the main factors affecting their participation in SDM as it helped them express their own wishes, cope with the pressure and challenge of making decisions within a short time in complex situations, and improve their enthusiasm for decision-making.

In conversations about patients' condition and treatment goals, which include a lot of medical jargon, it was important to ensure that surrogates understood these professional vocabularies. By exhibiting empathy and control of the pace of conversation in their communication, physicians can improve surrogates' understanding of professional knowledge and achieve emotional resonance with them, thus making communication smoother and enhancing family members' participation in the decision-making process. Conversely, surrogates' active participation in the decision-making process would reduce if they feel that physicians do not pay enough attention to them and do not have enough time to communicate with them.

If surrogates have many friends and relatives, the primary decision-makers may seek their counsel or ask other healthcare workers for advice before reaching a decision. Although family and friends can facilitate the decision-making process, disagreements among family members can delay the process. Many surrogates believed that peer support can better prepare patients for SDM.

In the decision-making process, value clarification was a process of identifying pros and cons, weighing the risks, and sorting the outcome-influencing factors by their importance. The treatment of choice had to align with what the patient would have wanted and preferred. In this process, physicians would actively inquire about and respect patients' wishes. Since most critically ill patients are not able to clearly express their values and preferences, without value clarification, it becomes difficult for doctors and surrogates to reach a consensus on the best treatment strategy and make correct decisions in line with the values and preferences of the patients. In critically ill patients, physicians often fully respect the will of patients and decide a treatment method consistent with patients' preferences after communication with surrogates.

Taken together, healthcare providers and surrogates shared the responsibility of making decisions. Surrogates reported that negotiation with healthcare providers often helped them reach a mutually agreeable decision, particularly for end-of-life decisions. In addition, because of the shift system in the ICU, healthcare providers change with changing shifts; this may limit healthcare providers' understanding of the needs of patients and their surrogates. Detailed briefing of the new staff about these needs during shift change can help physicians quickly understand the circumstances, and therefore, good medical service continuity between shifts is conducive to the implementation of SDM.

## 5. Discussion

This qualitative interview study explored the perspectives of the three stakeholders—ICU physicians, ICU nurses, and surrogates—on SDM. Similar to earlier studies, the concept of SDM has started gaining wide recognition, and most healthcare providers strongly acknowledged the significance of SDM [10, 15]. However, a few interviewees still did not clearly understand SDM and confused it with the traditional “informed consent model.” In particular, to some extent, nurses lacked clarity regarding their roles and responsibilities in SDM. ICU nurses of domestic hospitals rarely participated in SDM [16]. Similarly, surrogates do not yet understand the concept of SDM or its advantages. Therefore, they struggle with realizing the differences in their decision-making authority according to the gravity of patients' medical conditions; they also struggle with timely decision-making under high-pressure situations. The implementation of SDM needs to be based on the participation of both healthcare providers and surrogates. Some previous studies show that the traditional Chinese culture greatly influences surrogates' decision-making approach; they prefer to play a passive role in decision-making and wish for physicians to decide for them ([17]; Y. D. [18]). Thus, healthcare providers should correct this erroneous approach of surrogates and encourage them to actively contribute to the decision-making process.

In total, the three stakeholders focus on the end-of-life decision as the main decision for which SDM should be implemented. This study found that the surrogates struggled with making end-of-life decisions, which is in agreement with a previous report [5]. In terminal cases, the surrogates felt a sense of loss, anxiety, and denial, thus compromising their mental clarity for making a decision. Some surrogates could not accept the current treatment results of the patients and descended into a mindset of self-reproach; they often had a contradictory and obfuscating outlook toward their own decisions. Although it is widely recognized that SDM involves healthcare providers and surrogates reaching a consensus on a responsible decision, these decisions often involve lesser participation of and inputs from surrogates, particularly in families with inadequate educational levels [19]. Therefore, it is necessary to discuss the barriers and facilitators of the implementation of SDM.

This study identifies several barriers obstructing seamless implementation of SDM in the ICU setting. Based on the interview responses, we identified heavy workload and insufficient communication time of healthcare providers as obstacles affecting the implementation of SDM. In a previous study, insufficient communication time and interruption of intervention were identified as major obstacles faced by ICU healthcare providers for implementing SDM [20]. Lots of research institutions are constantly refining the implementation process of SDM and developing different decision aid tools. In China, using decision aids for patients on long-term mechanical ventilation, researchers helped the surrogates better comprehend medical knowledge and reported that this interaction reduced surrogates' decision-making dilemmas and uncertainty caused by anxiety, depression, and other symptoms (B. B. [21]). Presently, the SDM process is not standardized and localized decision aids are unavailable in China. Hospitals should draw learnings from foreign theoretical frameworks (e.g., Ottawa Decision Support Framework) which develop a robust implementation process for SDM, clearly define the core functions of healthcare providers in SDM, and develop decision aids that would be suitable for the Chinese population and medical system. Furthermore, the ability of healthcare providers to convey relevant theoretical knowledge to surrogates and patients' families in a simplified manner should be improved, which will reduce their work burden, improve the decision-making readiness of the family, and shorten the decision time.

This study identified several facilitators of SDM in the ICU setting. A previous study emphasized that ICU nurses should be involved in SDM [22]. Truglio et al. reported that owing to their rich clinical experience, ICU specialist nurses can contribute to SDM by guiding the surrogates with their decision-making process [23]. Nurses with longer and richer medical experience can better comprehend the psychological condition of patients and their families. Extending psychological support to patients' families helps SDM implementation by encouraging decision-makers to communicate and express their emotions. In routine care, caregivers should be empathetic, listen actively, and provide basic guidance with sufficient expertise in key areas of concern to the patient/family, including diet, complications, restraints, and skin-related issues. Supplementing verbal communication with reliable printed information leaflets or web-based decision aids is recommended. When surrogates are concerned about problems beyond the scope of nurses' expertise, the nursing staff should abridge the communication gap between physicians and surrogates to convey the perspective of surrogates to the physicians, thus optimizing the quality of nursing and improving the satisfaction of surrogates.

## 6. Study Limitations

Since the study includes a small sample size recruited from only one ICU of one hospital, the results may not be generalizable to all healthcare providers and surrogates. Nevertheless, the inclusion of different types of healthcare providers and surrogates offered a broad perspective on SDM, wherein we also identified consistent perspectives among the stakeholders regarding the perceived barriers and facilitators of SDM. Notwithstanding, additional (implementation) studies are needed to address these barriers and facilitators to improve the practice of SDM.

## 7. Conclusions

In the ICU, reaching treatment decisions is critical to proper medical management. It affects the patient's health outcomes and treatment experience. The necessary steps should be taken to implement SDM in a manner that is satisfactory to both agents and healthcare providers. Thirty participants (11 agents, 12 ICU physicians, and 7 ICU nurses) were interviewed. The three stakeholders showed different attitudes toward SDM. Based on this, we explored the attitudes of surrogates and health care providers toward SDM and identified the barriers and promoters of SDM in this population. In addition, this study also explored the different attitudes of the three stakeholders and found out various obstacles and promoting factors of SDM. It highlights the need to develop localised decision AIDS and to involve agents and nurses more in the decision-making process. Finally, we established the barriers and facilitators of SDM. The whole paper shows that the development of localised decision AIDS and greater involvement of agents and nurses in the decision-making process are integral to good treatment outcomes.

In the future, we hope to strengthen the attitudes and culture of both doctors and patients toward SDM. The medical side needs to accept the differences between the views of patients and medical staff and accept the questions of patients, so as to promote the SDM on the patient side and the public side. We also hope that people will understand that they are the owners of their own bodies and are responsible for their own health. It is not only a patient's right to express or ask questions to medical staff but also a duty to promote a positive medical environment through the joint efforts of both patients and doctors.

### 7.1. Relevance for Clinical Practice

SDM is currently in its infancy in ICU in China. To explore and clarify the barriers and facilitators affecting the implementation of SDM will help medical staff understand expectations of doctor-patient communication and decision-making from the perspective of surrogates and contribute to the promotion and application of SDM in clinical practice. This paper identifies barriers and facilitators of SDM in this population. In addition, the study identified various barriers and facilitators to SDM and highlighted the need to develop localized decision AIDS and involve agents and nurses more in the decision-making process. Finally, the barriers and facilitators of SDM are established. The paper shows that the development of localized decision AIDS and greater involvement of agents and nurses in the decision-making process are integral to good treatment outcomes.

## Figures and Tables

**Table 1:** Surrogate characteristics.

Interview order	Relationship with patient	Age	Gender	Highest education level
F1	Child of patient	47	Male	High school or less
F2	Parents of patient	58	Male	High school or less
F3	Brother of patient	30	Male	Associate's or Bachelor's degree
F4	Child of patient	42	Female	High school or less
F5	Grandchild of patient	32	Female	Associate's or Bachelor's degree
F6	Spouse of patient	31	Male	Associate's or Bachelor's degree
F7	Child of patient	41	Male	High school or less
F8	Son-in-law	54	Male	High school or less
F9	Child of patient	59	Male	High school or less
F10	Parents of patient	42	Female	High school or less
F11	Child of patient	49	Male	High school or less

**Table 2:** Healthcare provider characteristics.

Interview order	ICU physicians and nurses	Age group	Sex
D1	Intensivist	30–35	Female
D2	Intensivist	35–40	Female
D3	Intensivist	35–40	Female
D4	Intensivist	30–35	Female
D5	Intensivist	35–40	Female
D6	Intensivist	30–35	Female
D7	Intensivist	30–35	Female
D8	Intensivist	50–55	Male
D9	Intensivist	30–35	Male
D10	Intensivist	40–45	Male
D11	Intensivist	40–45	Male
D12	Intensivist	30–35	Female
N1	Intensive care nurse	30–35	Male
N2	Intensive care nurse	30–35	Male
N3	Intensive care nurse	30–35	Female
N4	Intensive care nurse	20–25	Female
N5	Intensive care nurse	25–30	Female
N6	Intensive care nurse	30–35	Female
N7	Intensive care nurse	40–45	Female

**Table 3:** Theme 1: different attitudes toward SDM.

Subtheme	Codes	Quotes
Physicians' supporting attitudes	“Decision-making requires collaboration,” “SDM is conducive to alleviating doctor-patient conflicts,” and “making decisions with surrogates”	D6: In clinical practice, I understand that it would be better to have more SDM because in the current treatment environment, doctors will take into account the values and various factors of the patient's family, and thus, SDM will be more suitable. If I am only responsible for conveying simple information and let the family members make their own choices, this would just be a communication. However, we also play a guiding role wherein we explain professional knowledge to patients and help them make decisions with their family members. D2: The choice of family members must be respected, but the conflict between doctors and patients is very serious, particularly for patients admitted to the ICU, and the family members have to make critical decisions regarding whether to intubate and whether to continue rescuing patients. We can only give suggestions, and SDM is good. D8: SDM is good, just like communication, which will help a lot. The main problem is that in China, communication is still not standardized.
Nurses' inconsistent attitudes: Supporting and affirming	“SDM is helpful,” “nurses are 24 hours at patients' bedside,” and “cooperation with doctors and families”	N1: I have heard of SDM. It can help doctors learn more about the patients' wishes. N7: We spend the most time at the patient's bedside and know what the patient is thinking.
Hesitating and doubting	“Lack of time” and “physician may ignore nurses' advice”	N4: At present, we still get informed consent signed by the patient or their surrogate, which prevents many conflicts between doctors and family members associated with any unfavorable outcome. How to implement SDM? Will there be a lot of trouble?” N5: If all clinical decisions need to be shared, it must take a lot of time; we are usually so busy, and there is often not enough time for this approach.
Surrogates' ambivalent attitudes: Willingness to participate in SDM	“Knowing what is coming and feeling included,” “more information means better outcomes,” and “feeling confident and secure”	F5: The doctor helped us make decisions and explained each treatment plan clearly. We also had a thorough understanding of the next treatment, which made us feel more secure about the treatment outcomes. F6: I think I can participate in the decision-making and make decisions by myself. After all, it is my relative who is admitted to the hospital. Although the doctor is also very important, I can feel relieved if I decide on my own.
No perceived need for SDM	“No attention for the family” and “lacking a feeling of control”	F9: You can decide whether to insert or not (endotracheal intubation) according to your professional expertise. F11: Although you explained everything, we cannot understand exactly what you were saying about surgery. We do not know what decide based on this information. We just have to accept what you are saying, right?

**Table 4:** Theme 2: barriers of SDM.

Subtheme	Codes	Quotes
Inadequate cognition of decision-makers	“Expecting doctors to make decision,” “be an obedient patient,” and “doctors are more professional”	F1: There's nothing I can do; it is up to you to save us. We do not understand this stuff. We do not know what you are talking about. We just agree with your treatment. After all, doctors are the most professional. We trust doctors. F6: Because we are unprofessional and doctors are professional, the doctors of course do the right thing. Because we are not professionals, we do not know much about it, but the doctors are doing the right thing. N2: Most family members do not have medical knowledge. When they go to the hospital, they have to follow the doctor's advice; some of them only know a little about it from the Internet, and that's even worse.
High expectation	“Hope to be cured,” “not give up,” and “do our best to try”	F2: We want the doctor to give us a clear treatment plan and explain in detail how the treatment is going to work. What is it going to take to cure him? F5: My message is very clear—as long as she has a breath, we must hold on. N4: Take the current bed 9 for example. We all know it is hard to cure him, but if the family members do not give up, there is nothing we can do.
Negative psychological experience	“Struggle to make decision,” “feel little hope and confused,” “fear a loss of control”	F3: I really do not know, I was quite emotional at the time, I did not read it carefully, and I forgot what I said. I'm so nervous, I'm so worried, I cannot remember what we talked about. F10: I forgot a little bit. To tell you the truth, I was also a little emotional at that time. I must have been worried about the children being sent here, and I also forgot the main details I talked about at that time.
Previous decision-making experience	“Have admitted to ICU before,” “heard the bad news,” and “without confidence to make decision”	F5: My dad was admitted to your ICU once; he had high creatinine, and he was there for a long time. Earlier, he was younger, so he came back, but now he cannot control himself. You tell him to drink less, but he cannot control himself. F7: Yesterday, I was in a bad mood because an old man in our family had an endotracheal tube inserted and died during extubation. I do not know what the problem was. So, this is a place that jangles my nerves. When the doctor called me and asked if he should intubate, I said no.
Excessive workload	“Doctors are too busy,” “the medical system does not support SDM,” and “too much work limits the conversation about treatment”	F3: Doctors are busy, and SDM takes too much time. F7: It can be difficult to find a doctor sometimes because the system is different. We looked for the doctor and waited a long time for a consultation; the door opened and we were told that the doctor was busy. Then, he told us to wait for a while. Sometimes the doctor came, and sometimes the busy doctor forgot. N5: Every morning from 9:00 to 12:00, a lot of treatment and basic care tasks are ongoing; there is no time to do this. I feel it is not possible to incorporate SDM in ICUs in China.
Financial burden	“Cannot afford the treatment,” “have to give up the treatment because of money problems”	D1: For example, financial problems. Some family members feel they can no longer support themselves financially, so they discontinue treatment. D2: For example, a patient who has not urinated needs to undergo hemodialysis, which is associated with high treatment costs. If the family cannot bear the financial pressure, they have to opt for diuretics or other solutions. N3: Some decisions for patients are obviously good, but they come with some financial difficulties. In fact, everyone loves their family, and they all want to get the best treatment for their family members, but some people, after all, are limited by their economic condition, which is one of the biggest factors for treatment discontinuation, and some people may also not have that much time and energy.
Lack of decision aids	“Appropriate tools make decision easier” and “lack the aids to make decision”	D5: Sometimes you talk to family members for a long time, but they still do not know what you are talking about. It's just a waste of time, and there are no appropriate tools in clinical practice. N4: For example, for deep vein catheterization and endotracheal intubation, the family members do not know what kind of tube it is and how thick it is. How can they make decisions? N6: If there are pictures or some simple, easy-to-understand animations of procedures performed in clinical practice, they can be understood by family members at a glance and will facilitate smoother conversations during SDM.

**Table 5:** Theme 3: facilitators of SDM.

Subthemes	Codes	Quotes
Trust	“Trust comes from healthcare providers' professional level,” “trust facilitates SDM,” and “trust makes communication smoother”	D4: Patients' trust comes from your understanding of their condition and professional level, which is the most important factor for patients to trust you the first time. Only after they trust you can they speak freely with you and effectively make shared decisions with you. N6: The final decision is a matter of trust in doctors. Family members trust doctors, and thus, they can communicate with each other easily, and the treatment will be much smoother. On the other hand, because of access to unverified medical media on the internet that is presented as factually correct information, some medical disputes are exaggerated, which lead to the tension between doctors and patients. F2: I'm sure we trust you, and that's why we are here. We were prepared before we came to the ICU, so we gave it a try.
Effective communication	“Control the pace of conversation” and “put yourself in the patient's shoes”	D1: In short, it is important to reach a state wherein two people can sympathize with each other. Sometimes we are talking about our professional knowledge, but the family members cannot understand it completely. So, the ability to empathize is important. The other thing, which is about keeping a humane approach, is that when talking about an illness, we often try to control the pace in which the information is conveyed based on the family's ability to process and understand the information, and thus, the pace is very important. D12: First, I think I should be professional in my conduct and the judgment of the illness. In addition, I can put myself in the other's shoes. From the point of view of family members, I can understand their psychological condition and communicate better accordingly.
Decision support	“Decision support from others,” “suggestions from friends, family and healthcare providers”	F2: I consulted family members before making a decision. It is a big deal. Who would think of drinking like that at a young age? After talking to them, I feel more confident. F4: My family has been discussing it for two or three days. Now we basically know the cause of the disease and the condition. We have made a good decision according to the situation. N5: Even my neighbors sometimes ask my opinion on whether there is a need for hospitalization.
Value clarification	“The doctor gave full consideration to the patient's opinions,” “doctors seek the patient's preferred treatment,” and “respect the patient's opinion”	D5: Yes, it is also related to his (a family member's) views. If the family member is very active, the doctor will be more active and take active measures because there is no one way to save the patient's life for sure. F9: Doctors also asked our family members for our opinions. They respected our opinion. N4: In fact, sometimes I think I have thought on behalf of the family members, but we are not family members. Although we can try our best to think for them, we may never be able to feel for them as much as a family member would. Everybody's situation is different, and everybody's family dynamics are different, right?
Outcome commitment	“Stopping treatment is a shared choice” and “accept the results together”	F4: We've been debating for days whether to send him home or not. He was awake earlier and spoke with us clearly, but now his condition is worsening; we tried our best, but him passing away seems likely. We made this decision, and we accept the results and are willing to bear with the outcome. We know that the doctors did their best and thank them for it. F7: Actually, to be honest, at first thought, you come to the hospital to cure people, right? But even after all efforts, if there is no way to recover from this disease, we have to accept that. This requires the doctor to clearly communicate with us and speak without being obscure so that we can prepare ourselves to bear any result.
Continuous service	“Shift change,” “handover of special circumstances,” and “understand details”	D1: We will do a detailed shift on the patient's condition, willingness of family members and communication problems. This ensures that doctors on shift or on weekends are getting consistent information as well.

## Data Availability

The datasets used and analyzed during the current study are available from the corresponding author upon reasonable request.

## Additional Points

*Key Points*. (1) Shared decision-making (SDM) approach is seldom adapted in the ICU, so the purpose of this study is to explore the barriers and facilitators of SDM from the perspectives of surrogates and healthcare providers. (2) The implementation of ICU SDM is complicated, and there are both hindering and promoting factors. Developing localized decision aids and greater inclusion of surrogates and nurses in the decision-making process are necessary for the implementation of SDM. (3) This study comprehensively understands the decision-making process between surrogates and healthcare providers in ICU and provides theoretical basis for the construction of localized ICU shared decision-making model.
